The article "EBV Promotes Human CD8+ NKT Cell Development" was retracted in 2010. Reasons: fabricated or falsified images; concerns about the images; concerns about the results or conclusions.

# EBV Promotes Human CD8^+^ NKT Cell Development

**DOI:** 10.1371/journal.ppat.1000915

**Published:** 2010-05-20

**Authors:** He Yuling, Xiao Ruijing, Ji Xiang, Li Li, Chen Lang, Xiong Jie, Xiao Wei, Wang Yujuan, Zhang Lijun, Zhou Rui, Tan Xinti, Bi Yongyi, Jiang Yan-Ping, Jin Youxin, Tan Jinquan

**Affiliations:** 1 Department of Immunology, Wuhan University School of Medicine, Wuhan, People's Republic of China; 2 Laboratory of Allergy and Clinical Immunology, Institute of Allergy and Immune-related Diseases, Centre for Medical Research, Wuhan University School of Medicine, Wuhan, People's Republic of China; 3 Section of Geriatrics, Departments of Internal Medicine, The Renmin University Hospital, Wuhan University, Wuhan, People's Republic of China; 4 Wuhan University School of Public Health, Wuhan, People's Republic of China; 5 The State Key Laboratory of Molecular Biology, Institute of Biochemistry and Cell Biology, Shanghai Institutes for Biological Sciences, Chinese Academy of Science, Shanghai, People's Republic of China; Indiana University School of Medicine, United States of America

## Abstract

The reports on the origin of human CD8^+^ Vα24^+^ T-cell receptor (TCR) natural killer T (NKT) cells are controversial. The underlying mechanism that controls human CD4 versus CD8 NKT cell development is not well-characterized. In the present study, we have studied total 177 eligible patients and subjects including 128 healthy latent Epstein-Barr-virus(EBV)-infected subjects, 17 newly-onset acute infectious mononucleosis patients, 16 newly-diagnosed EBV-associated Hodgkin lymphoma patients, and 16 EBV-negative normal control subjects. We have established human-thymus/liver-SCID chimera, reaggregated thymic organ culture, and fetal thymic organ culture. We here show that the average frequency of total and CD8^+^ NKT cells in PBMCs from 128 healthy latent EBV-infected subjects is significantly higher than in 17 acute EBV infectious mononucleosis patients, 16 EBV-associated Hodgkin lymphoma patients, and 16 EBV-negative normal control subjects. However, the frequency of total and CD8^+^ NKT cells is remarkably increased in the acute EBV infectious mononucleosis patients at year 1 post-onset. EBV-challenge promotes CD8^+^ NKT cell development in the thymus of human-thymus/liver-SCID chimeras. The frequency of total (3% of thymic cells) and CD8^+^ NKT cells (∼25% of NKT cells) is significantly increased in EBV-challenged chimeras, compared to those in the unchallenged chimeras (<0.01% of thymic cells, CD8^+^ NKT cells undetectable, respectively). The EBV-induced increase in thymic NKT cells is also reflected in the periphery, where there is an increase in total and CD8^+^ NKT cells in liver and peripheral blood in EBV-challenged chimeras. EBV-induced thymic CD8^+^ NKT cells display an activated memory phenotype (CD69^+^CD45RO^hi^CD161^+^CD62L^lo^). After EBV-challenge, a proportion of NKT precursors diverges from DP thymocytes, develops and differentiates into mature CD8^+^ NKT cells in thymus in EBV-challenged human-thymus/liver-SCID chimeras or reaggregated thymic organ cultures. Thymic antigen-presenting EBV-infected dendritic cells are required for this process. IL-7, produced mainly by thymic dendritic cells, is a major and essential factor for CD8^+^ NKT cell differentiation in EBV-challenged human-thymus/liver-SCID chimeras and fetal thymic organ cultures. Additionally, these EBV-induced CD8^+^ NKT cells produce remarkably more perforin than that in counterpart CD4^+^ NKT cells, and predominately express CD8αα homodimer in their co-receptor. Thus, upon interaction with certain viruses, CD8 lineage-specific NKT cells are developed, differentiated and matured intrathymically, a finding with potential therapeutic importance against viral infections and tumors.

The article "EBV Promotes Human CD8+ NKT Cell Development" was retracted in 2010. Reasons: fabricated or falsified images; concerns about the images; concerns about the results or conclusions.

## Author Summary

We show that the average frequency of total and CD8^+^ NKT cells in PBMCs from 128 healthy latent EBV-infected subjects is significantly higher than in 17 patients with acute lytic EBV infection, 16 EBV-associated HL patients, and 16 EBV-negative normal subjects. The frequency of total and CD8^+^ NKT cells is remarkably increased in the lytic EBV-infected patients at year 1 post-onset. EBV-challenge promotes total and CD8^+^ NKT cell development in the thymus and liver of human-thymus/liver-SCID chimeras, compared to those in the unchallenged chimeras. After EBV-challenge, a proportion of NKT precursors diverges from DP thymocytes, develops and differentiates into mature CD8^+^ NKT cells in thymus in EBV-challenged human-thymus/liver-SCID chimeras or reaggregated thymic organ cultures. Thymic EBV-infected dendritic cells are required for this process. IL-7 is an essential factor for CD8^+^ NKT cell differentiation. EBV-induced CD8^+^ NKT cells produce remarkably more perforin, and predominately express CD8αα homodimer. CD8 lineage-specific NKT cells are developed and differentiated intrathymically upon EBV-exposure, a finding with potential therapeutic importance against viral infections and tumors.

## Introduction

NKT cells are unconventional T cells that bridge the innate and adaptive immune systems [1]–[4]. Unlike conventional T cells, which recognize MHC-molecule-presented peptide antigens via their αβTCR, NKT cells recognize CD1d-presented glycolipids. Two subsets of functionally distinct CD1d-dependent NKT cells have been identified based on whether the cells express the semi-invariant Vα24-Jα18 TCR (Vα14-Jα18 in mice) [1], [2], [5]–[12] and whether they recognize the exogenous NKT cell ligand α-GalCer. Other NKT-like cells have been reported based on their CD1d-independence and CD161 (NK1.1 in mouse) or CD56 expression [12]–[16], or other semi-invariant Vα7.2-Jα33/Vβ2,13 TCR expression (Vα19/Vβ6,8 in mouse) [12].

The article "EBV Promotes Human CD8+ NKT Cell Development" was retracted in 2010. Reasons: fabricated or falsified images; concerns about the images; concerns about the results or conclusions.

In mice, conventional αβT cell development in the thymus proceeds through three major stages, i.e. CD4^−^CD8^−^ (DN), CD4^+^CD8^+^ (DP), and CD4^+^CD8^−^ or CD4^−^CD8^+^ (SP) [17]. The developing αβT cells undergo positive and negative selection based on TCR affinity of MHC expressed on antigen presenting cells. By contrast, the semi-invariant αβTCR DP NKT precursors interact with the CD1d-ligand complex either on cortical thymocytes to undergo positive selection [1]–[2], or on thymic dendritic cells (DCs) to undergo negative selection [18]. Positively selected DP NKT cell precursors mature by down-regulating CD8 to reach a CD4^+^CD44^lo^ stage [1]–[2]. Unlike conventional T cells, which emigrate from the thymus as naïve cells, CD44^lo^ NKT cells remain in the postnatal thymus and undergo a linear differentiation program including the expression of the terminal differentiation marker NK1.1 [19], [20]. However, a proportion of the immature NKT cells remains NK1.1^−^ and leaves the thymus [19], [20]. The final NKT-differentiation step takes place in both thymus and periphery [21], [22]. Peripheral NKT cells reside preferentially in the liver [23], [24], but are also present in the spleen, lymph nodes, bone marrow, lung, and gut [1], [2]. Human NKT cells have not been detected in engrafted fetal thymus tissue in a hu-thy/liv-SCID model, leading to a presumption that the development of peripheral NKT cells is thymus independent [25]. In later studies, it was proposed that the human thymus has little or no role in generating peripheral NKT cells after birth. This hypothesis is based on the inverse correlation between NKT cell frequency in fetal thymus and gestational age, and on the lack of a clear NKT cell population in postnatal thymus but their definite presence in adult blood [26]–[28]. However, reports on the origin of human CD8^+^ Vα24^+^TCR NKT cells are still controversial.

In mice, it is believed that there are essentially no CD8^+^ NKT cells [1], [2], [29]. However, recent report shows that IL-15 expands CD8ααNK1.1^+^ cells [30]. In humans, the existence of CD8^+^ NKT cells in thymus and periphery is an area of controversy. CD8^+^ αβTCR NKT cells expressing CD8αα homodimer are reported in human PBMC [31]. While there are several reports questioning the existence of these cells [26], [32], it is widely believed that CD8 is expressed on a minor proportion of human NKT cells, and that the CD8 marker is usually acquired after egress from the thymus [27], [28], [33]–[37]. The finding of a limited correlation between human thymic CD4^+^ NKT cells and peripheral CD8^+^ NKT cells has raised the question of what is the origin of CD8^+^ NKT cells [27], [28]. As accumulation of findings on NKT cell development, the underlying mechanisms that control CD4-CD8 differentiation of human NKT cells are becoming better characterized.

The article "EBV Promotes Human CD8+ NKT Cell Development" was retracted in 2010. Reasons: fabricated or falsified images; concerns about the images; concerns about the results or conclusions.

## Results

### EBV-induced CD8^+^ NKT cells in various EBV-infected individuals

We studied 177 eligible patients and subjects including 128 healthy latent EBV-infected subjects [EBV^+^(La)], 17 newly-onset acute infectious mononucleosis patients [EBV^+^(IMa)], 16 newly-diagnosed EBV-associated Hodgkin lymphoma patients [EBV^+^(HL)], and 16 EBV-negative normal control subjects (NS) (Table S1). None of the individuals had received treatment with anti-virals, antibiotics, or corticosteroids before entry into this study. The race of all individuals was Han as determined and registered by the physicians in this study. None of the individuals had other complicating clinical infectious symptoms when the study samples were taken. The average frequency of total NKT cells in PBMCs from the 128 EBV^+^(La) subjects (1.5±0.5%) was significantly higher than that from 16 EBV-negative NS subjects (0.18±0.2%), 17 new-onset EBV^+^(IMa) patients (0.15±0.1%) and 16 newly-diagnosed EBV^+^(HL) patients (0.1±0.1%) (Figure 1B). The frequency of total NKT cells in the EBV^+^(IMa) patients dramatically increased at year 1 post-onset [EBV^+^(IMy), 1.6±0.6%] (Figure 1B). The frequency of the CD8^+^ subset of NKT cells in PBMCs from the EBV^+^(La) subjects (17±4%) was remarkably higher than from EBV-negative NS subjects (2.1±0.3%), new-onset EBV^+^(IMa) patients (1.9±0.4%) and EBV^+^(HL) patients (1.1±0.2%) (Figure 1B). The frequency of CD8^+^ NKT cells in the EBV^+^(IMa) patients was significantly increased at year 1 post-onset [EBV^+^(IMy), 20±5%] (Figure 1B). However, the average frequencies of total T cells and the ratios of CD4^+^ versus CD8^+^ T cells in PBMCs among the EBV^+^(La), EBV^+^(HL), EBV^+^(IMy) and NS subjects were not significantly different (Figure 1C), except for a slight and temporary increase in the frequency of total T cells in the EBV^+^(IMa) patients (Figure 1C, some data not shown). These observations clearly indicate that the EBV status affects the frequency of NKT cells, particularly, the appearance of CD8^+^ NKT cells in PBMC.

**Figure 1:** Human NKT and T cells in the various EBV-infected and non-infected subjects. (**A**) The experimental and analysis scheme for detecting co-receptor-expressing NKT cells and T cells in PBMC was illustrated. The data to establish negative staining gates with fluorochrome conjugated empty CD1d tetramers (eCD1d tetramer) and αβTCR isotype mAb (αβTCRIso) control was shown in rightmost panel of this subfigure. (**B**) and (**C**) Frequencies of total (left panel) and co-receptor-expressing (right panel) NKT (**B**) and conventional αβT cells (**C**) in PBMCs from healthy latent EBV-infected subjects [EBV^+^(La)], newly-onset acute infectious mononucleosis patients [EBV^+^(IMa)], IM patients at year 1 post-onset [EBV^+^(IMy)], EBV-associated HL patients [EBV^+^(HL)] and EBV-negative normal control subjects (NS) assessed by flow cytometry. The absolute numbers per ml of NKT cell subsets of various patient and subject were shown in bottom panel as means ± s.d. (the s.d. was not shown for simplicity of the figure) (**B**). Data were mean ± s.d. (For patient numbers see Table S1). *, *p*<0.001.

The article "EBV Promotes Human CD8+ NKT Cell Development" was retracted in 2010. Reasons: fabricated or falsified images; concerns about the images; concerns about the results or conclusions.

### EBV induces intrathymic CD8^+^ NKT cell development

To investigate the mechanism of total and CD8-lineage differentiation of human NKT cells in the context of EBV, we established hu-thy/liv-SCID chimeras. The chimeras were challenged i.t. with EBV, a dsDNA virus, or with human T-cell leukaemia virus type 1 (HTLV-1), a retrovirus. The EBV-challenge efficiently promoted the generation of total NKT cells, whereas HTLV-1-challenge had no effect, but instead promoted a significant increase in the frequency of αβTCR thymocytes and spleen T cells (Figure 2A). The frequency of total NKT cells reached more than 3% of thymic cells and more than 2% of hepatic cells by week 5 post-challenge with EBV. By contrast, the total thymic and hepatic NKT cells were less than 0.01% within 5 weeks post-challenge with HTLV-1, comparable to the frequencies in unchallenged chimeras (Figure 2A). The frequencies of total thymic or hepatic T cells at week 5 were slightly but significantly increased following HTLV-1 infection. There were approximately 30,000–35,000 total NKT cells per million thymic cells, and 20,000–23,000 total NKT cells per million hepatic cells at week 5 in EBV-challenged chimeras (Table S2). The EBV-challenge did not significantly alter the generation of total mainstream αβT cells, whereas HTLV-1-challenge did promote the generation of the T cells, compared with those in unchallenged chimeras (Figure 2B). The frequency of total T cells reached ∼28% of thymic cells and ∼32% of spleen cells at week 5 in the chimeras challenged with EBV or HTLV-1, as well as in the unchallenged chimeras (Figure 2B). Cell phenotyping based on CD4 and CD8 expression (Figure 2C) revealed that EBV-challenge significantly promoted the generation of thymic CD8^+^ NKT cells and the appearance of hepatic CD8^+^ NKT cells in the chimeras transplanted i.t. with total thymocytes (NKT cell-depleted) plus thymic stromal cells, a population that includes DC (Figure 2E), compared to unchallenged chimeras (Figure 2D). By contrast, HTLV-1-challenge had no effect on the frequency of CD8^+^ NKT cells (data not shown). The frequency of CD8^+^ cells in the chimeras reached more than 25% of thymic NKT cells and more than 23% of hepatic NKT cells at week 5 post-EBV challenge (Figure 2E). The CD8^+^ cells were essentially undetectable among thymic and hepatic NKT cells at 5 weeks in the unchallenged chimeras (Figure 2D). The different thymic or hepatic NKT cell populations (DN, CD4^+^, and CD8^+^) in the HTLV-1-challenged chimeras were comparable to those in the unchallenged chimeras (data not shown). The frequencies of total and CD4/CD8 co-receptor-expressing NKT cells in peripheral blood correlated well with those in thymus and livers in both unchallenged and EBV-challenged hu-thy/liv-SCID chimeras (data not shown). An important role for DCs in the generation of thymic and hepatic CD8^+^ NKT cells is suggested by the finding that the frequency of these cells was rather low in both unchallenged and EBV-challenged chimeras transplanted i.t. with total fetal thymocytes plus DC-depleted thymic stromal cells (data not shown), an issue explored further below. The different thymic and spleen co-receptor-expressing mainstream T cells (DN, CD4^+^CD8^lo^, CD4^+^, CD8^+^) in the EBV- or HTLV-1-challenged chimeras were comparable to those in the unchallenged chimeras (Figure 2D, 2E, and some data not shown). The absolute numbers of NKT cells and αβT cells (thymocytes) in the organs from various hu-thy/liv-SCID chimers were shown in the Table S2.

The article "EBV Promotes Human CD8+ NKT Cell Development" was retracted in 2010. Reasons: fabricated or falsified images; concerns about the images; concerns about the results or conclusions.

**Figure 2:** EBV promotes CD8^+^ NKT cell development *in vivo* in hu-thy/liv-SCID chimeric mice. (**A**) and (**B**) Development of total NKT (**A**) and T cells (**B**). The frequencies of NKT cells and T cells in thymus, liver, and spleen from hu-thy/liv-SCID chimeras challenged i.t. with EBV (EBV^+^) or HTLV-1 (HTLV-1^+^), were assessed by flow cytometry (middle and right panels) at the indicated timepoints. Unchallenged hu-thy/liv-SCID chimeras (Nil) were used as controls. Empty CD1d tetramer and isotype matched control Abs, which were used as staining controls, were not illustrated in this figure. The experimental and analysis scheme was shown in the leftmost panel. Data were mean ± s.d. (n  =  8). *, *p*<0.001. EBV-challenged chimeras vs. non-challenged or HTLV-1-challenged chimeras. (**C**) The experimental and analysis scheme for detecting the co-receptor-expressing NKT cells and T cells in various organs from different hu-thy/liv-SCID chimeras was illustrated. The α-GalCer-loaded CD1d tetramer, αβTCR mAb and other relevant mAbs were used to identify the different subsets of NKT cells and T cells as illustrated. The appropriate isotype Abs and empty fluorochrome-conjugated CD1d tetramer were used as controls. (**D**) and (**E**) Data showed the frequencies of co-receptor-expressing NKT cells and T cells in the unchallenged (**D**, Nil) or EBV challenged (**E**, EBV) hu-thy/liv-SCID chimeras. The protocols for the establishment of the chimeras were described in the leftmost panels. The chimeras were sacrificed at the indicated time intervals following post-immune-reconstitution and viral challenge and the various organs and tissues were collected. +DC, thymic DCs were included. VL, very low level (below detectable levels). Data were mean ± s.d. (n  =  7). *, *p*<0.001, EBV-challenged chimeras vs. non-challenged or HTLV-1-challenged chimeras.

Thymic CD8^+^ NKT cells from EBV-challenged hu-thy/liv-SCID chimeras displayed an activated memory phenotype (CD69^+^CD45RO^hi^), compared with thymic CD4^+^ NKT cells in same chimeras (Figure S1A). Hepatic CD8^+^ NKT cells expressed higher amounts of CD62L than thymic CD8^+^ NKT cells in the EBV-challenged chimeras, probably attributable to their egress from the thymus toward secondary lymphoid organs, whereas these hepatic CD8^+^ NKT cells expressed similar amounts of CD69 and CD45RO as thymic CD8^+^ NKT cells (data not shown). CD161, a maturation marker for human NKT cells, was uniformly highly expressed on thymic and hepatic CD8^+^ NKT cells in EBV-challenged chimeras; the frequency of CD8^+^ NKT cells in the unchallenged chimeras was too low to evaluate CD161 expression. On CD4^+^ NKT cells, CD161 expression was independent of EBV challenge and revealed two populations, CD161^hi^ and CD161^lo^, although the former population expressed much higher levels of CD161 in the EBV treated mice (Figure S1A and some data not shown). In parallel, we also examined the expression of CD69, CD62L and CD45RO on thymic and spleenic CD4^+^, CD4^+^CD8^lo^, CD4^+^CD8^+^, and CD8^+^ T cells in EBV-challenged or unchallenged chimeras. Both CD4^+^ and CD8^+^ T cells in thymus and spleen from EBV-challenged hu-thy/liv-SCID chimeras displayed an activated memory phenotype (CD69^+^CD45RO^hi^), compared with T cells from unchallenged chimeras (Figure S2B and some data not shown). Spleen CD4^+^ and CD8^+^ T cells in EBV-challenged chimeras expressed higher amounts of CD62L (data not shown) than the thymic CD4^+^ and CD8^+^ T cells (Figure S1B), which might be attributable to their egress from the thymus to secondary lymph organs.

The article "EBV Promotes Human CD8+ NKT Cell Development" was retracted in 2010. Reasons: fabricated or falsified images; concerns about the images; concerns about the results or conclusions.

### EBV-induced CD8^+^ NKT cell development depends on thymic DCs

We established different hu-thy/liv-SCID chimeras by i.t. transplantation with purified human fetal DP thymocytes plus thymic stromal cells (either DC-containing or DC-depleted). In chimeras transplanted DN thymocytes only, the frequency of total NKT cells was very low (<0.01% of thymic or hepatic cells) at week 5 in both unchallenged and EBV-challenged mice (Figure 3B, 3C). The great majority of cells were CD4-expressing in both chimeras. Less than 0.5% of thymic and hepatic CD8^+^ NKT cells were detected in EBV-challenged chimeras (Figure 3C). Both the frequency of total αβTCR-expressing T cells and the ratio of CD4^+^ to CD8^+^ T cells in thymus and spleen from EBV-challenged hu-thy/liv-SCID chimera transplanted with DP thymocytes only (Figure 3B, 3C) were comparable to those in EBV-challenged or unchallenged chimeras transplanted with total thymocytes (Figure 2). We further examined the ontogeny and distribution of NKT cells and T cells in hu-thy/liv-SCID chimeras transplanted i.t. with fetal DP thymocytes plus DC-containing thymic stromal cells. The frequency of total NKT cells was still rather low (∼0.02% of thymic or hepatic cells) at week 5 post-establishment in the unchallenged chimeras (Figure 3D), but was substantially increased (∼3% of thymic or hepatic cells) at week 5 post-establishment in EBV-challenged chimeras (Figure 3E). Up to 25% of thymic or hepatic NKT cells expressed CD8 in EBV-challenged chimeras, whereas the frequencies of thymic or hepatic CD4^+^ NKT cells were correspondingly lower than those in the unchallenged chimeras (Figure 3D, 3E). The frequency of total mature αβTCR-expressing T cells and the ratio of CD4^+^ to CD8^+^ T cells in thymus and spleen in EBV-challenged hu-thy/liv-SCID chimeras were comparable to those in unchallenged chimeras (Figure 3D, 3E). The development of thymic or hepatic CD8^+^ NKT cells was severely impaired by the DC-deletion. The frequency of thymic and hepatic CD8^+^ NKT cells was essentially below the level of detection in both unchallenged and EBV-challenged chimera transplanted i.t. with DP thymocytes plus DC-depleted thymic stromal cells (Figure 3F, 3G). We also examined the ontogeny and distribution of NKT cells and T cells in the hu-thy/liv-SCID chimeras transplanted i.t. with DP thymocytes plus purified thymic DC. The frequency of total thymic and hepatic NKT cells and the ratio of CD4^+^ to CD8^+^ NKT cells in EBV-challenged or unchallenged chimeras were comparable to those in the counterpart chimeras transplanted with DP thymocytes plus DC-included thymic stromal cells (data not shown). We further established hu-thy/liv-SCID chimeras by transplantation i.t. with fetal DP thymocytes plus i.v. syngeneic fetal BM-derived DCs. The frequency of total NKT cells was substantially increased to ∼2% of thymic or hepatic cells at week 5 post-establishment in the EBV-challenged chimeras (Figure 3I), compared to the unchallenged chimeras (∼0.01% of thymic or hepatic cells) (Figure 3H). Up to 23% of thymic and hepatic NKT cells expressed CD8 in the EBV-challenged chimeras, whereas the levels of thymic and hepatic CD4^+^ NKT cells were correspondingly lower than those in the unchallenged chimeras (Figure 3H, 3I). The frequency of total mature αβTCR-expressing T cells and the ratio of CD4^+^ to CD8^+^ T cells in thymus and spleen from EBV-challenged hu-thy/liv-SCID chimeras were comparable with those in the unchallenged chimeras (Figure 3H, 3I). The absolute numbers of NKT cells and αβT cells (thymocytes) in the organs from various hu-thy/liv-SCID chimers were shown in the Table S2.

The article "EBV Promotes Human CD8+ NKT Cell Development" was retracted in 2010. Reasons: fabricated or falsified images; concerns about the images; concerns about the results or conclusions.

**Figure 3:** EBV-induced CD8^+^ NKT cell development occurs at the DP thymocyte stage and depends upon thymic dendritic cells. (**A**) The experimental and analysis scheme for detecting co-receptor-expressing NKT cells and T cells in various organs from different hu-thy/liv-SCID chimeras is illustrated after collecting 2.0×10^6^ total cell events. (**B**–**I**) Development of co-receptor-expressing NKT cells (middle panels) and T cells (right panels). Data illustrate the frequency of co-receptor-expressing NKT cells and T cells in thymus, liver and spleen from EBV-challenged hu-thy/liv-SCID chimeras (EBV). Unchallenged hu-thy/liv-SCID chimeras (Nil) were used as controls. The protocols for the establishment of the various hu-thy/liv-SCID chimeras were described in the leftmost panels. (**B**–**G**) Instead of total thymocytes, hu-thy/liv-SCID chimeras were established by intrathymic transplantation with DP thymocytes. The chimeras were sacrificed at the indicated time points following post-immune-reconstitution and viral challenge. Staining was performed as in Figure 2. +DC, thymic DCs were included. -DC, thymic DCs were depleted. In (**H**) and (**I**) the hu-thy/liv-SCID chimeras were established by intrathymic transplantation with DP thymocytes. Instead of transplantation with thymic stromal cells, BM-derived dendritic cells (1×10^6^ cells) were injected i.v. into the hu-thy/liv-SCID chimeras at t = 0. VL, very low level (below detectable level). ND, no determination. Data (**B**–**I**) were mean ± s.d. (n  =  8). *, *p*<0.001, EBV-challenged chimeras vs. non-challenged chimeras.

The article "EBV Promotes Human CD8+ NKT Cell Development" was retracted in 2010. Reasons: fabricated or falsified images; concerns about the images; concerns about the results or conclusions.

We next performed various RTOC of human fetal DP thymocytes reaggregated with syngeneic fetal thymic stromal cells (thymic DC-included), purified thymic DCs, or BM-derived DCs. Various stimuli (EBV-epitopes, infectious EBV or α-GalCer) were applied during the culture. The frequency of total NKT cells was low (<0.01% of RTOC cells) in the EBV- or α-GalCer-challenged RTOC established with only DP thymocytes (Figure 4B). In RTOC of DP thymocytes reaggregated with syngeneic fetal thymic stromal cells (thymic DC-included), purified thymic DCs, or BM-derived DCs, the EBV-challenge significantly promoted the generation of total NKT cells. After 14-day-culture, the frequency of total NKT cells was up to 2.5–2.8% of RTOC cells, whereas treatment with α-GalCer had no such effect (Figure 4B). Addition of HLA-matched or unmatched EBV-epitopes (BMLF1+EBNA1) had no significant effect on the frequency of total NKT cells (<0.01% of RTOC cells) compared to the un-stimulated RTOC (Figure 4B and data not shown). In RTOCs where thymic or BM-derived DCs were present, EBV-challenge substantially promoted the development of CD8^+^ NKT cells. Up to 25% of NKT cells expressed CD8 in EBV-challenged RTOCs (Figure 4C). In this case, HLA-matched EBV-epitopes moderately and significantly increased the development of CD8^+^ NKT cells (2.5% of NKT cells), compared with those in un-stimulated RTOCs (Figure 4C). In RTOC of DP thymocytes reaggregated with DC-depleted thymic stromal cells, the EBV-induced increase in CD8^+^ NKT was almost completely abolished (data not shown). Both the frequency of total mature αβTCR-expressing T cells and the ratio of CD4^+^ to CD8^+^ T cells in the different RTOC conditions were comparable (Figure 4B, 4D).

**Figure 4:** EBV-induced CD8^+^ NKT cell differentiation depends upon thymic dendritic cells. (**A**) The experimental and analysis scheme for detecting co-receptor-expressing NKT cells and T cells in various reaggregated fetal thymic organ cultures (RTOCs). After 14-days of culture, the various cell types were identified by flow cytometry as in Figure 2. (**B**–**D**) Frequency of total NKT cells and total T cells (**B**), co-receptor-expressing NKT cells (**C**) and T cells (**D**), in the different RTOCs. The protocols for the establishment of the RTOCs were described in the leftmost panels in each sub-figure: DP thymocytes were reaggregated with either total thymic stromal cells (DC-included), purified thymic dendritic cells, or BM-derived dendritic cells. The stimuli were added as indicated. Nil, no stimulus; EBV-epitopes, HLA-A2-restricted, derived from the lytic cycle protein BMLF1 and HLA-DRB1-restricted, derived from nuclear antigen EBNA1 (10 µg/ml each); EBV, infectious EBV (10^7^ pfu); Solvent, 0.005% polysorbate 20; α-GalCer (0.1 µg/ml). The RTOCs were harvested, and assessed by flow cytometry. Only the data for CD4^+^ and CD8^+^ NKT cells, and CD4 SP and CD8 SP T cells were shown. VL, very low level (below detectable level). Data were mean ± s.d. (n  =  10). *, *p*<0.001, EBV-challenged RTOCs vs. non-challenged RTOCs.

The article "EBV Promotes Human CD8+ NKT Cell Development" was retracted in 2010. Reasons: fabricated or falsified images; concerns about the images; concerns about the results or conclusions.

To further confirm that EBV mediated intrathymic CD8-lineage differentiation of human NKT cells, we focused our attention on detecting the actual EBV- or HTLV-1-infection of human progenitor thymocytes, thymic NKT cells and thymic DCs in the virus exposed hu-thy/liv-SCID chimeras. For detection of EBV-infection, five transformation-associated EBV-genes, LMP1, EBNA1, BZLFl, BALF2, and RAZ were examined. By Southern blot and Q-PCR, a high level of viral genes and mRNA transcripts were detected in EBV-exposed human DCs in the chimeras. Since mice are not the natural EBV host and their DCs are well-known to be unsusceptible to EBV, these results indicated that EBV infected only the transplanted human DCs in EBV-exposed hu-thy/liv-SCID chimeras during NKT cell development and differentiation. There was no evidence of EBV viral genes in EBV-exposed human chimeric DP thymocytes or mature CD4^+^ and CD8^+^ NKT cells (Figure S2A). For detection of HTLV-1-infection, 2 highly conserved viral X-region DNA sequences, SK43 and SK44, were examined. By Q-PCR assay, high levels of SK43 and SK44 were detected in human chimeric HTLV-1-exposed DP αβTCR-expressing T cells (Figure S2B) as well as in chimeric hepatic T cells (data not shown). There was no detectable HTLV-1 in thymic CD4^+^ and CD8^+^ NKT cells or in DCs in the HTLV-1-exposed hu-thy/liv-SCID chimeras, indicating that HTLV-1 virus does not correlate with NKT cell differentiation in EBV-exposed hu-thy/liv-SCID chimeras.

### EBV-induced CD8^+^ NKT cell development is IL-7-dependent

IL-7 and IL-15 were known survival factors for T cells, and enhancers of NKT cell homeostatic proliferation [21], [26], [38], [39]. Both cytokines were used in attempts to differentiate and activate NKT cells from human peripheral and cord blood [35], [40], [41]. DP thymocytes expressed an increased level of IL-7Rα in EBV-challenged hu-thy/liv-SCID chimeras compared to unchallenged chimeras. The thymic DCs produced a considerable amount of IL-7 mRNA in unchallenged chimeras, and the levels increased substantially with EBV-challenge (Figure S3A). The thymic CD8^+^ NKT cells expressed a very high level of IL-7Rα mRNA in EBV-challenged hu-thy/liv-SCID chimeras compared with other types of thymic NKT cells and αβTCR-expressing T cells in both unchallenged and EBV-challenged chimeras (Figure S3A). The thymic DCs produced a considerable amount of IL-15 mRNA in both unchallenged and EBV-challenged chimeras. The thymic CD4^+^ and DN NKT cells expressed higher levels of IL-15Rα mRNA in both unchallenged and EBV-challenged hu-thy/liv-SCID chimeras compared with other types of thymic NKT cells and αβTCR-expressing T cells in both chimeras (Figure S3A). In a time course study, the freshly isolated fetal thymic DCs were found to express a low level of IL-7 mRNA. Thymic DCs in unchallenged chimeras expressed comparable levels of IL-7 mRNA at the different time intervals examined, 1, 3, and 5 weeks. By contrast, the thymic DCs rapidly increased the expression of IL-7 mRNA by week 1 post-EBV challenge, and maintained high levels throughout the course of the analysis (Figure S3B). The IL-15 mRNA was uniformly expressed in the thymic DCs of both unchallenged and EBV-challenged chimeras (Figure S3B). Thymic stromal cells (DC-depleted) expressed a uniformly low level of IL-7 and IL-15 mRNA in both unchallenged and EBV-challenged chimeras (data not shown). These observations on cytokine and cytokine receptor mRNA expression were confirmed at the protein level by intracellular flow cytometry (for IL-7 and IL-15) and conventional flow cytometry (for IL-7Rα and IL-15Rα) (data not shown). Thus, the thymic DCs are a major source of IL-7 during the thymus-dependent development of NKT cells.

The article "EBV Promotes Human CD8+ NKT Cell Development" was retracted in 2010. Reasons: fabricated or falsified images; concerns about the images; concerns about the results or conclusions.

The frequency of total NKT cells were low (<0.01% of FTOC cells) after 14-days of culture without adding any stimuli in FTOC (Figure 5B). Nearly all of the NKT cells were CD4-positive and CD8^+^ cells were undetectable in these conditions (Figure 5C). By contrast, in FTOC with added EBV, the frequency of total NKT cells was increased (1.5% of FTOC cells), and of these, 15% of cells expressed CD8, whereas, in FTOC with added HLA-matched EBV-epitopes, neither total nor CD8^+^ NKT cells were changed (<0.01% of FTOC cells, of which <1% were CD8^+^) (Figure 5C). Exogenous IL-7 or IL-15 alone slightly but significantly increased the total, but not CD8^+^ NKT cell differentiation in the FTOCs (<0.01% of FTOC cells) (Figure 5C). HLA-mismatched EBV-epitopes were non-functional in FTOCs (data not shown). In EBV-challenged FTOCs, exogenous IL-7, but not IL-15, could significantly further enhance the total and CD8^+^ NKT cell differentiation (∼2.5% of FTOC cells, of which 20% were CD8^+^), compared to the EBV-challenged but non-IL-7-stimulated FTOC and un-stimulated FTOC (Figure 5B, 5C). A mAb against IL-7 completely abolished the effect of IL-7 on the differentiation of CD8^+^ NKT cells in the EBV-challenged FTOCs, indicating an essential role of the cytokine in the differentiation of CD8^+^ NKT cells. In FTOCs containing added α-GalCer, IL-7 slightly enhanced total, but not CD8^+^ NKT cell differentiation (∼1% of FTOC cells, of which <0.8% were CD8^+^) (Figure 5B, 5C). The mAb against IL-7 completely inhibited the effect of IL-7 on the differentiation of total NKT cells in the FTOCs stimulated with α-GalCer. IL-15 had no such effect on the development of total NKT cells in the FTOCs stimulated with α-GalCer. The frequency of total mature αβTCR-expressing T cells, but not ratios of CD4^+^ to CD8^+^ T cells, was enhanced by IL-7 or/and IL-15 in the various FTOCs (Figure 5B, 5C).

The article "EBV Promotes Human CD8+ NKT Cell Development" was retracted in 2010. Reasons: fabricated or falsified images; concerns about the images; concerns about the results or conclusions.

**Figure 5:** IL-7 is required for EBV-induced CD8^+^ NKT cell differentiation *in vitro*. (**A**) The experimental and analysis scheme for detecting co-receptor-expressing NKT cells and T cells in various human fetal thymic organ cultures. After 14-day-culture, the various cell types were identified by flow cytometry as in Figure 2. (**B**–**D**) Frequency of total NKT cells and total T cells (**B**), co-receptor-expressing NKT cells (**C**) and T cells (**D**) in the different FTOCs. The protocols for the establishment of different FTOCs were described in the leftmost panels in each sub-figure. The various stimuli and blockers were added as indicated. Nil, no stimulus; EBV-epitopes, HLA-A2-restricted, derived from the lytic cycle protein BMLF1 and HLA-DRB1-restricted, derived from nuclear antigen EBNA1 (1 µg/ml each); EBV, infectious EBV (10^7^ pfu); Solvent, 0.005% polysorbate 20; α-GalCer (0.1 µg/ml). IL-7 (10 ng/ml); IL-15 (10 ng/ml), Abs, either mouse anti-human IL-7 monoclonal Ab plus mouse anti-human IL-7Rα monoclonal Ab, or mouse anti-human IL-15 monoclonal Ab plus mouse anti-human IL-15Rα monoclonal Ab, respectively (5 µg/ml each); The FTOCs were harvested and assessed by flow cytometry. Only the data for CD4^+^ and CD8^+^ NKT cells and CD4 SP and CD8 SP T cells were shown. VL, very low level (below detectable level). Data were mean ± s.d. (n = 10). ** *p*<0.05. *, *p*<0.001, EBV-challenged FTOCs vs. non-challenged FTOCs; IL-7-challenged FTOCs vs. non-challenged FTOCs.

Consistent with the above *in vitro* findings in the FTOCs, administration of exogenous IL-7 further enhanced development of thymic and hepatic total and CD8^+^ NKT cells in the *in vivo* EBV-challenged hu-thy/liv-SCID chimeras (Figure 6B), compared to chimeras given exogenous IL-7 but not EBV (data not shown) and to EBV-challenged chimeras not treated with exogenous IL-7 (Figure 2E). The frequency of total NKT cells was significantly increased (∼3.8% of thymic and ∼3.2% hepatic cells) (Figure 6B). About 28% of thymic and hepatic NKT cells expressed CD8 (Figure 6B and Table S2). The administration of mAb against IL-7 (plus exogenous IL-7) completely blocked the function of IL-7 *in vivo* (Figure 6C and Table S2), indicating an essential role of the cytokine in the EBV-induced development of CD8^+^ NKT cells. The administration of exogenous IL-7 plus isotype-matched control Ab had no the blocking effect (Figure 6D and Table S2). Thus, EBV-induced increase in CD8^+^ NKT cell development is IL7-dependent.

The article "EBV Promotes Human CD8+ NKT Cell Development" was retracted in 2010. Reasons: fabricated or falsified images; concerns about the images; concerns about the results or conclusions.

**Figure 6:** IL-7 is required for EBV-induced CD8^+^ NKT cell development *in vivo*. (**A**) The experimental and analysis scheme for detecting co-receptor-expressing NKT cells and T cells in various organs from hu-thy/liv-SCID chimeras treated with IL-7. The chimeras were established by intrathymic transplantation with DP thymocytes. The chimeras were treated i.v. with IL-7 (0.1 µg/kg/d), or with IL-7 plus mAb against IL-7 (1 µg/kg/d) (IL-7+Ab), or IL-7 plus isotype Ab (1 µg/kg/d) (IL-7+Iso) as indicated. The chimeras were sacrificed at the indicated time points following post-immune-reconstitution and viral challenge. Staining was performed as in Figure 2. (**B**–**D**) Development of co-receptor-expressing NKT cells. Data show the frequency of co-receptor-expressing NKT cells in thymus or livers from hu-thy/liv-SCID chimera challenged i.t. with EBV (EBV), as assessed by flow cytometry. The protocols for the establishment of the chimeras were described in the leftmost panel. +DC, thymic DCs were included. VL, very low level (below detectable level). Data (**B**–**D**) were mean ± s.d. (n = 7 or 8). *, *p*<0.001, EBV- and IL-7-challenged chimeras vs. a-IL-7 Ab-treated chimeras.

To track NKT cells more accurately, we applied 6B11 mAb, which recognized TCR Vα24JαQ junction CDR3-loop, combined with mAb against Vα24TCR for gate of NKT cells by flow cytometry. The outcome of frequencies of total and co-receptor-expressing NKT cells gated by either CD1d tetramers vs. anti-αβTCR mAb or by anti-Vα24 mAb vs. 6B11 mAb were comparable in different human normal subjects or EBV-infected patients (Figure S4A). Comparable sets of data on frequencies of total and co-receptor-expressing NKT cells were also obtained in thymus and liver from EBV-challenged hu-thy/liv-SCID chimeras (Figure S4B), as well as in EBV-exposed RTOCs and FTOCs (data not shown), gated by either CD1d tetramers vs. anti-αβTCR mAb or anti-Vα24 mAb vs. 6B11 mAb by flow cytometry. These data confirmed the observations on EBV-induced development of CD8^+^ NKT cells, and ruled out possible contamination of activated conventional CD8^+^ T cells during the flow cytometry analysis.

### EBV-induced CD8^+^ NKT cells produce abundant perforin

In our recent study [42], frequencies of CD8^+^ NKT cells in patients with EBV-associated malignancies were found significantly lower than those in healthy EBV carriers. CD8^+^ NKT cells in tumor patients were functionally impaired in terms of cytokine production and cytotoxicity. In hu-thy/liv-SCID chimeras, EBV-exposure efficiently augmented the generation of IFN-γ-biased CD8^+^ NKT cells, which were strongly cytotoxic to EBV-associated tumor-cells. IL-4-biased CD4^+^ NKT cells were predominately generated in unchallenged chimeras, which were non-cytotoxic. In tumor-transplanted hu-thy/liv-SCID chimeras, adoptive transfer with EBV-induced CD8^+^ NKT cells remarkably suppressed tumorigenesis by EBV-associated malignancies. CD4^+^ NKT cells were synergetic with CD8^+^ NKT cells, leading to a more pronounced T-cell anti-tumor response in the chimeras co-transferred with CD4^+^ and CD8^+^ NKT cells. In the present study, we further investigated the perforin expression in NKT cells (Figure 7). CD8^+^ NKT cells from healthy EBV^+^ humans, EBV-challenged hu-thy/liv-SCID chimeras, or EBV-exposed RTOCs and FTOCs produced much higher amount of perforin (Figure 7B) than that in counterpart CD4^+^ NKT cells (Figure 7A), indicating that high production of perforin in EBV-induced CD8^+^ NKT cells was an additional reason for their high cytotoxicity to EBV-associated tumor cells, besides their biased IFN-γ-production [42]. In the analysis, we applied flow cytometry using the gating of either CD1d tetramers vs. anti-αβTCR mAb and anti-Vα24 mAb vs. 6B11 mAb. Two groups of results were comparable (Figure 7).

The article "EBV Promotes Human CD8+ NKT Cell Development" was retracted in 2010. Reasons: fabricated or falsified images; concerns about the images; concerns about the results or conclusions.

**Figure 7:** Perforin expression in human and chimeric CD4^+^ and CD8^+^ NKT cells. PBMC were from healthy latent EBV-infected subjects [EBV^+^(La)], IM patients at year 1 post-onset [EBV^+^(IMy)], EBV-associated HL patients [EBV^+^(HL)] and EBV-negative normal control subjects (NS). Thymic cell suspension were from EBV-exposed (EBV^+^), un-exposed (EBV^−^) or HTLV-1-exposed (HTLV-1^+^) hu-thy/liv-SCID chimeras, or from EBV-exposed (EBV^+^) or un-exposed (EBV^−^) RTOC and FTOC. For detection of intracellular expression of perforin, cells were stimulated with α-GalCer (1 µg/ml) for 24 hrs, intracellular stained, and assessed by flow cytometry using the experimental strategy shown in the upper panel of each subfigure. The NKT cells were gated by either CD1d tetramers vs. anti-αβTCR mAb (middel panels) or anti-Vα24 mAb vs. 6B11 mAb (bottom panels). Perforin positive cells (%) in gated CD4^+^ (**A**) and CD8^+^ (**B**) NKT cells were shon. Solvent for α-GalCer was 0.005% polysorbate 20 (not shown). Nil, negative stimulation control. ND, no determination. Data were mean ± s.d. (n = 8). **, p<0.05; *, p<0.001. CD8^+^ in (**B**) vs. counterpart CD4^+^ NKT cells in (**A**).

The article "EBV Promotes Human CD8+ NKT Cell Development" was retracted in 2010. Reasons: fabricated or falsified images; concerns about the images; concerns about the results or conclusions.

Moreover, we further analyzed the CD8α and CD8β expression on NKT cells. Data revealed that CD8αα homodimer was predominately expressed on CD8^+^ NKT cells in PBMCs from healthy latent EBV-infected subjects and IM patients at year 1 post-onset, as well as from normal control subjects (Figure 8B and 8C), which were consistent with the previous reports [31]. CD8αα homodimer was also expressed in the majority of CD8^+^ NKT cells in thymus and liver from hu-thy/liv-SCID chimeras challenged i.t. with EBV (Figure 8D and 8E) and in EBV-exposed RTOCs and FTOCs (data not shown). In the analysis, we applied flow cytometry using the gating of either CD1d tetramers vs. anti-αβTCR mAb and anti-Vα24 mAb vs. 6B11 mAb. Two groups of results were comparable (Figure 8).

**Figure 8:** NKT cells differentially express the CD8α and CD8β chain. (**A**) The experimental and analysis scheme for detecting total and co-receptor CD8α- and CD8β-expressing NKT cells. (**B**) and (**C**) NKT cells in PBMCs from healthy latent EBV-infected subjects [EBV^+^(La)], IM patients at year 1 post-onset [EBV^+^(IMy)], EBV-associated HL patients [EBV^+^(HL)] and EBV-negative normal control subjects (NS) were assessed by flow cytometry using the gate of either CD1d tetramers vs. anti-αβTCR mAb (**B**) or anti-Vα24 mAb vs. 6B11 mAb (**C**). Further dot plot analysis of CD8α vs. CD8β in gated NKT cells was shown. (**D**) and (**E**), NKT cells in thymus (Thy) and liver (Liv) from hu-thy/liv-SCID chimeras challenged i.t. with EBV (EBV^+^) or unchallenged (EBV^−^) were assessed by flow cytometry using the gate of either CD1d tetramers vs. anti-αβTCR mAb (**D**) or anti-Vα24 mAb vs. 6B11 mAb (**E**). Further dot plot analysis of CD8α vs. CD8β in gated NKT cells was shown. Data were representatives of 5 similar experiments in each group.

## Discussion

Taken advantage of the hu-thy/liv-SCID chimeric mouse model [43], [44], we have found that a sizable CD8^+^ fraction (up to 25%) of total human thymic NKT cells is generated *in vivo* after EBV-challenge. The development of CD8^+^ NKT cells is promoted in the thymus at the DP precursor stage, and requires participation of thymic DCs. CD4 versus CD8 lineage commitment is controlled by the EBV-challenge. The findings provide a crucial access point for unraveling the mechanism for NKT cell development and differentiation. This study led to two important insights. First, we provide direct evidence that certain pathogens, EBV in this case, are important contributors to CD8-lineage commitment of NKT cells. Second, we demonstrate that differential CD4 versus CD8 lineage commitment can be controlled not only by some known classical endogenous elements [1], [2], but also by exogenous pathogenic element(s) such as EBV.

The article "EBV Promotes Human CD8+ NKT Cell Development" was retracted in 2010. Reasons: fabricated or falsified images; concerns about the images; concerns about the results or conclusions.

The impact of different viral pathogens on NKT cell frequencies has been investigated. In humans, infection by HIV and HTLV-1 results in a decrease in NKT cells [45]–[52]. In mice, LCMV induces long-term loss of NKT cells since induction of apoptosis [53], [54]. The patients with severe immunodeficiency (XLP), lacking of NKT cells, is characterized by an extreme sensitivity to EBV infection [55], [56]. Our previous [42] and current works show that EBV-infection promotes generation of IFN-γ- and perforin-biased CD8^+^ NKT cells, and IL-4-biased CD4^+^ NKT cells. A protective role of CD8^+^ NKT cells synergized with their counterpart CD4^+^ NKT cells against EBV-associated malignancies has been verified. The beneficial role against the persistence of EBV-infection could be speculated. The observation on induction of dominate populations of CD8αα^+^ NKT cells by EBV-infection is in agreement with previous report on that CD8αα^+^ NKT cells control expansion of total and EBV-specific T cells in humans [31], and is supporting the observation in mice [30].

There remain several controversial issues concerning CD8^+^ NKT cell development. For example, why does the frequency of human CD8^+^ NKT cells show such a limited correlation between different sites (thymus and blood) and among different ages (fetus, neonate and adults), and why are CD8^+^ NKT cells the most numerically variable NKT cell subset in humans, particularly under pathophysiological circumstances [1], [2], [26]–[28], [33]–[37]. In the present study, we were able to monitor the intrathymic and extrathymic development of human NKT cells in different organs in hu-thy/liv-SCID chimeric mice. Since all mature NKT cells were depleted from the thymocytes prior to cell transplantation (Figure S6), any co-receptor-expressing human NKT cells detected in the mice should have developed and differentiated post-cell-transplantation. Since all fetal samples have been from non-EBV-infected mothers, the EBV-challenge in this animal model accurately reflects the viral effects on the differentiation of CD8^+^ NKT cells. Nevertheless, more evidences are needed to rule out the possibility that EBV is capable of influencing NKT cell expansion/differentiation in the periphery.

Given the functional distinction between CD4^+^ and CD8^+^ NKT cells [26]–[28], [33]–[37] and their potential therapeutic importance such as in cancer treatment [42], it is crucial to identify the factors that induce the development and differentiation of these cells in order to fully understand the causes of NKT cell subset deficiency and dysfunction, particularly of the CD8^+^ NKT cells. Some investigators hold the opinion that the immature NKT cells undergo extrathymic differentiation in adult blood [27], [28], [33]–[37]. Our studies have demonstrated that the frequency of total NKT cells and the different subsets in thymus, liver and peripheral blood from unchallenged and EBV-challenged chimeras is highly correlated, clearly indicating an intrathymic developmental and differentiation step for human CD8^+^ Vα24^+^NKT cells. Moreover, the hu-thy/liv-SCID chimeras have provided an *in vivo* model to investigate cell development and differentiation of human NKT cells under both physiological and pathophysiological circumstances.

The article "EBV Promotes Human CD8+ NKT Cell Development" was retracted in 2010. Reasons: fabricated or falsified images; concerns about the images; concerns about the results or conclusions.

In mice, IL-15 plays an essential role in the maturation and overall population size of NKT cells in the thymus and periphery [21], [22], [30]. On the other hand, IL-7 is critical for the development of NKT cells, but plays a minor role in regulating their maturation and homeostasis [21]. In humans, IL-7 dominates the CD4^+^ NKT cell development process in the fetus, neonate, and adult [26], [39], whereas IL-15 has a selective and age-specific role *in vitro* in the expansion and homeostasis of the DN and CD8^+^ NKT cell subsets [27]. We show here that IL-7 is a major and essential enhancer of EBV-induced development of thymic CD8^+^ NKT cells *in vivo*, in the hu-thy/liv-SCID chimeras, and *in vitro* in FTOCs. We still need to define the role of IL-7 in the continuous NKT cell division in the periphery of adults, if it indeed exists, for instance, in secondary lymphoid organs where IL-7 is available.

Taking the fact that EBV causes asymptomatic life-long infection in ∼90% of adults worldwide into consideration, the experimental design for developmental studies of NKT cells should pay special attention to the EBV status of the donors of any human samples, since we have shown here that EBV-infection status of the hu-thy/liv-SCID chimeras and the human donors can directly affect the frequency of total and co-receptor-expressing populations of NKT cells. More importantly, the present study has raised several interesting questions, such as how the semi-invariant canonical αβTCR is expressed on DP thymocyte precursor before commitment to the CD4 versus CD8 lineage differentiation of NKT cells, as well as what and how the ligand is presented by thymic DCs to the semi-invariant αβTCR-expressing DP thymocyte precursor causing the preferential CD8 differentiation.

## Materials and Methods

### Patients, cells, tetramers, and other reagents

The latent EBV-infected [referred to as EBV^+^(La)] or normal control subjects (NS) were healthy EBV seropositive or seronegative individuals, respectively. The patients with EBV-associated acute infectious mononucleosis [lytic phase, referred to as EBV^+^(IMa)] were diagnosed by a monospot test and the detection of capsid-specific serum IgM [56], and followed-up at 1 year [latent phase, referred to as EBV^+^(IMy)]. The patients with EBV-associated Hodgkin lymphoma (HL) were diagnosed according to the WHO criteria, and staged according to the Ann Arbor classification (Table S1). All EBV^+^(La) and NS individuals were healthy volunteers. All patients eligible for this study were in- or out-patients in different Hospitals in Hubei Province in China. HLA typing was performed using the Lymphotype Class I system (Biotest) and an Olerup SSP kit (GenoVision). The clinical information of all patients and healthy EBV-infected and normal control subjects is listed in Table S1. All patients were newly-diagnosed and had no previous treatment before entry into this study. All patients provided informed consent according to the institutional guidelines and protocol titled “The study on the frequency and subset distributions of human peripheral NKT cells in normal and EBV-infected subjects” that was approved by The Wuhan University Ethical Committee. The written informed consent from each patients and subjects was obtained.

The article "EBV Promotes Human CD8+ NKT Cell Development" was retracted in 2010. Reasons: fabricated or falsified images; concerns about the images; concerns about the results or conclusions.

Human fetal thymic cells, bone marrow (BM) cells, liver and PBMCs were anonymously obtained from voluntarily elective pregnancy terminations (<24-wk-gestation; HLA typing matched HLA-A2 and HLA-DRB1(*03), the most prevalent HLA-types for Eastern and Southern Chinese populations, and mismatched HLA-A11, -B8 and HLA-DQ5). The mothers were excluded if lytic and latent EBV- and HTLV-1-infections were detected by Q-PCR and serologic determination [57]. Thymic cells, BM cells and PBMCs were isolated, aliquoted, cryopreserved and maintained in the vapor phase of liquid nitrogen for further use. Viability of thawed cells was evaluated by Trypan blue dye exclusion before use. Thymic dendritic cells were separated from the thymocytes by adhesion onto plastic culture dishes. For transplantation, NKT cells were positively depleted from thymic cells by MACS beads based on staining with α-GalCer-loaded CD1d tetramers [58]. For functional studies, NKT cells were purified from human PBMCs or chimeric thymic cells by flow cytometry cell sorting or a MACS bead system based on staining with α-GalCer-loaded CD1d tetramers [58], [59]. Synthesized peptides (proteins) were EBV-epitopes, GLCTLVAML (HLA-A2-restricted, derived from the lytic cycle protein BMLF1), AVFDRKSDAK (HLA-A11-restricted, derived from nuclear antigen EBNA3B), RAKFKQLL (HLA-B8-restricted, derived from the lytic cycle protein BZLF1), TSLYNLRRGTAL (HLA-DRB1-restricted, derived from nuclear antigen EBNA1), SDDELPYIDPNM (HLA-DQ5-restricted, derived from nuclear antigen EBNA3C) [60]. Recombinant peptides (proteins) were verified free of pyrogenicity (endotoxin <10 units/ml, no bacterial or fungal contamination) according to the certifications from the manufacturer. The α-GalCer-loaded CD1d tetramers were synthesized as previously described [58]–[60]. For preparation of viral stocks, a highly productive EBV-producer cell line P3HR-1 (American Type Culture Collection, ATCC, Manassas, VA) was treated with 12-*O*-tetradecanoyl-phorbol-13-acetate (TPA, 30 ng/ml) for 14 days. The virus was then pelleted from the culture supernatant. The residual TPA in the viral suspension for final use had no significant promoting effect on cell proliferation in the *in vivo* human-thymus-SCID chimeras, based on our preliminary experiments. Recombinant human (rh) IL-7 (Roche) and rhIL-15 were purchased from R&D Systems. All mouse anti-human monoclonal antibodies were purchased from BD PharMingen, San Diego, CA, USA, except mAbs against human Vα24 or Vβ11, which were from Immunotech, Marseille, France.

The article "EBV Promotes Human CD8+ NKT Cell Development" was retracted in 2010. Reasons: fabricated or falsified images; concerns about the images; concerns about the results or conclusions.

### Human-thymus/liver-SCID chimeras

To establish the human-thymus/liver-SCID (hu-thy/liv-SCID) chimeras, 8-wk-old female SCID mice (NOD/LtSz-prkdc^scid^/prkdc^scid^ strain, the Jackson Laboratory) were irradiated (300 cGy/mouse) prior to cell-transplantation. Human fetal thymic cells were depleted of immature and mature NKT cells based on their reactivity with α-GalCer-loaded CD1d tetramers. Then, 1×10^7^ thymocytes, thymocytes: thymic stromal cells including dendritic cells = 1∶1 (Figure S5), were transplanted into the thymus of anaesthetized SCID mice [43], [44], [58], [59]. Syngeneic human fetal liver tissue (equivalent to 1×10^7^ fetal liver cells) was simultaneously implanted under the mouse kidney capsule, unless otherwise noted. The chimeras were then intrathymically challenged with EBV (10^7^ pfu) [60] or HTLV-1 (10^7^ pfu), and the challenge was repeated after 6 days. The chimeras were maintained for 4 wks, unless otherwise stated [43], [44]. In some cases, chimeras were established by transplantation with human fetal thymic cells (thymocytes plus thymic stromal cells), but without implantation of fetal liver tissue referred to as human-thymus-SCID (hu-thy-SCID chimera). The mice were housed in a pathogen-free environment in the Animal Research Institute, Wuhan University. The protocol for animal study titled “The study on the frequency and subset distributions of NKT cells in human-thymus/liver-SCID chimeras” was approved by The Wuhan University Ethical Committee in accordance with the current Chinese laws.

The article "EBV Promotes Human CD8+ NKT Cell Development" was retracted in 2010. Reasons: fabricated or falsified images; concerns about the images; concerns about the results or conclusions.

### Fetal thymic organ culture (FTOC) and reaggregated thymic organ culture (RTOC)

FTOC was carried out as described previously [61]. Briefly, fetal thymus tissue was dissected into pieces of ∼2 mm^3^. Three pieces of tissue were placed into 24-well plates with culture medium containing various stimuli as indicated. On day 7, the cultured thymus fragment was dispersed into a single-cell suspension, and cells were stained and analyzed by flow cytometry. RTOC experiments were performed as previously described [61]. Briefly, thymic stromal cells were prepared by disaggregating fetal thymic lobes. DP thymocytes were obtained by gently grinding freshly fetal thymus lobes. The resulting suspensions were sorted for DP thymocytes using CD4 and CD8 labeling. Reaggregates were formed by mixing together the desired thymic stromal cells and DP thymocytes at 1∶1 cell ratio with other stimuli as indicated. After pelleting the cells by centrifugation, the cell mixture was placed as a standing drop on the upper membrane surface, and incubated for 5–12 days.

### Flow cytometry

The α-GalCer-loaded CD1d tetramer and αβTCR (Immunotech, clone BMA031) was used to define total NKT cells. For tetramer staining, the cells were incubated with the tetramer labeled with fluorochromes at 37°C for 15 min. The appropriate isotype Ab (αβTCR mAb isotype mouse IgG_2b_) and empty CD1d tetramer conjugated with a fluorochrome was used to establish negative staining gates. The representative experiments for NKT cell gate negative staining were illustrated in Figure 1 and Figure S6. The αβTCR and other relevant mAbs were used to identify the different subsets of T cells. In some cases, mAb against human CDR3 loop of invariant TCR Vα24 (6B11, Immunotech) and mAb against human Vα24 (including isotype controls) were used for gating NKT cells. For analysis of co-receptor-expressing NKT cells, single cell suspensions were stained with mAbs to human CD4 and CD8α (R&D Systems, clone 11830 and 37006, isotype mouse IgG_2a_ and IgG_2b_), unless otherwise noted. In some cases, NKT cells were stained with mAbs to CD8α and CD8β (Abcam, clone 2ST8.5H7, isotype mouse IgG2a), simultaneously. In intracellular staining for detection of perforin, different cells were resuspended in cold Dulbecco's PBS, and then permeabilized by Cytofix/Cytoperm solution (15 min, 4°C, in the dark; BD Pharmingen) according to the manufacturer's protocol. These permeabilized cells were stained with mAb specific for human perforin (FITC-conjugated G9, mouse IgG_2b_, BD Pharmingen), or isotype control, and analyzed by flow cytometry. All analyses were performed with a FACSCalibur (BD Biosciences). Four- and five-color analysis was done using CellQuest software.

The article "EBV Promotes Human CD8+ NKT Cell Development" was retracted in 2010. Reasons: fabricated or falsified images; concerns about the images; concerns about the results or conclusions.

### Real time quantitative RT-PCR (Q-PCR)

All Q-PCR reactions were performed as described elsewhere [62]. Briefly, total RNA from purified cells (1×10^4^, purity >99%) or cell lines was prepared by using Quick Prep® total RNA extraction kit (Pharmacia Biotech) according to the manufacturer's instructions. RNA was reverse transcribed by using oligo (dT)_12-18_ and Superscript II reverse transcriptase (Life Technologies, Grand Island, USA). The real time quantitative PCR was performed in special optical tubes in a 96 well microtiter plate (Applied Biosystems, Foster City, CA) with an ABI PRISM® 7700 Sequence Detector Systems (Applied Biosystems). By using the SYBR® Green PCR Core Reagents Kit, fluorescence signals were generated during each PCR cycle via the 5′ to 3′ endonuclease activity of AmpliTaq Gold to provide real time quantitative PCR information. Primers used in Q-PCR are listed in Table S3.

### Statistical analysis

Statistical analyses were performed using the Student′s *t* test. Values of *p*<0.05 were considered statistically significant.

## Supporting Information

Figure S1 EBV-induced *in vivo* CD8^+^ NKT cells are mature and activated. Data showed the expression of CD69, CD45RO, CD62L, and CD161 on co-receptor-expressing NKT cells (**A**) and T cells (**B**) in thymus from the unchallenged (EBV^−^) or EBV challenged (EBV^+^) hu-thy/liv-SCID chimeras, as assessed by flow cytometry. The chimeras were sacrificed at week 5 of post-immune-reconstitution and viral challenge. The various organs and tissues were collected. The experimental and analysis scheme was illustrated in Figure 2. Empty fluorochrome conjugated CD1d tetramers were used as a staining control. ND, no determination since too few cells were detected. Data were representative of each of 5 sets of experiments conducted (n = 7).
(0.33 MB PDF)

Figure S2 EBV- or HTLV-1-infection of T cells, thymic NKT cells and dendritic cells from hu-thy/liv-SCID chimeras. The chimeras were challenged with either EBV (+) or HTLV-1 (+) for 4 weeks as described in M&M, or left un-challenged (−). The animals were then sacrificed. Human fetal primary (Prim.) thymocytes, total NKT cells or thymic NKT cells, and dendritic cells (DCs) in hu-thy/liv-SCID chimeras were purified according to the αβTCR and co-receptor expression, i.e. CD4^+^CD8^+^ (DP), CD4^−^CD8^−^ (DN), CD4^+^ and CD8^+^ cells. The different purified cells were washed extensively after purification. (**A**) Southern blot (top panel) and Q-PCR (bottom panel) analyses for detections of various EBV genomic DNA and mRNA transcripts, respectively. The primers and probes used were shown in Table S3. The applied methods were detailed in the references listed below [63], [64]. The EBV-transformed Raji B cell line (EBV^+^ B cell line) was used as a positive control. Data were representative (each n = 6). ND, no determination since too few cells harvested. For simplification, Q-PCR data from various cells were only shown for the representative EBV-exposed NP thymocytes, EBV-exposed CD4^+^ and CD8^+^ NKT cells, and EBV-exposed DCs. (**B**) Q-PCR detection of HTLV-1-infection in genomic DNA extract from various cells from HTLV-1-exposed (+) hu-thy/liv-SCID chimeras as described above. The HTLV-1 primer sets were designed corresponding to the highly conserved HTLV-1 pX region, referred to as SK43 (top panel) and SK44 (bottom panel) [65], [66]. The HTLV-1-infected T-cell lymphoma cell line HUT102 (HTLV-1^+^ T cell line) was used as a positive control. ND, no determination since too few cells harvested. Data were mean ± s.d. (n = 6).
(0.41 MB PDF)

Figure S3 EBV-challenge up-regulates IL-7 expression in thymic dendritic cells. (**A**) Expression of IL-7, IL-7 receptor alpha chain (IL-7Rα) (top panels), IL-15, and IL-15 receptor alpha chain (IL-15Rα) (bottom panels) mRNAs in different thymic cells. The hu-thy/liv-SCID chimeras were established by i.t. challenge with EBV (EBV^+^). Unchallenged hu-thy/liv-SCID chimeras (EBV^−^) were used as controls. The chimeras were sacrificed at week 5 post-immune-reconstitution and viral challenge. The indicated cell types were isolated and IL-7, IL-7Rα, IL-15, and IL-15Rα mRNA levels were assessed by Q-PCR. Data were mean ± s.d. (n = 8). *, *p*<0.001. (**B**) The time course study of IL-7 and IL-15 mRNA expression in thymic dendritic cells in different chimeras. The hu-thy/liv-SCID chimeras were established by i.t. challenge with EBV (EBV^+^). Unchallenged hu-thy/liv-SCID chimeras (EBV^−^) were used as a control. The chimeras were sacrificed at the indicated time points following immune-reconstitution and viral challenge. IL-7 and IL-15 mRNA levels were assessed by Q-PCR. Data were mean ± s.d. (n = 9). *, *p*<0.001, EBV-challenged chimeras vs. non-challenged chimeras.
(0.13 MB PDF)

Figure S4 Comparison among the outcomes of the frequencies of NKT cell subsets using two different gating staining by flow cytometry. The comparison was carried out between the counterpart frequencies of total and co-receptor-expressing NKT cells gated by either CD1d tetramers vs. anti-αβTCR mAb or by anti-Vα24 mAb vs. 6B11 mAb (anti-*i*TCR Vα24JαQ junction CDR3-loop). (**A**) The experimental and analysis scheme for detecting total and co-receptor-expressing NKT cells in PBMC was illustrated in upper panel. Frequencies of total (left subfigures) and co-receptor-expressing (right subfigures) NKT cells in PBMCs from healthy latent EBV-infected subjects [EBV^+^(La)], newly-onset acute infectious mononucleosis patients [EBV^+^(IMa)], IM patients at year 1 post-onset [EBV^+^(IMy)], EBV-associated HL patients [EBV^+^(HL)] and EBV-negative normal control subjects (NS) were assessed by flow cytometry using the gating by either CD1d tetramers vs. anti-αβTCR mAb (middle panels) or anti-Vα24 mAb vs. 6B11 mAb (bottom panels). Data were mean ± s.d. (n = 4). *, *p*<0.001. EBV^+^(La) or EBV^+^(IMy) vs, EBV^+^(IMa), NS or EBV^+^(HL). (**B**) The experimental and analysis scheme for detecting total and co-receptor-expressing NKT cells in thymus and liver was illustrated in upper panel. The frequencies of NKT cells in thymus and liver from hu-thy/liv-SCID chimeras challenged i.t. with EBV were assessed by flow cytometry at the indicated timepoints using the gating by either CD1d tetramers vs. anti-αβTCR mAb (left panel) or anti-Vα24 mAb vs. 6B11 mAb (right panel). Data were mean ± s.d. (n = 4). *, *p*<0.001. EBV^+^ vs. EBV^−^ hu-thy/liv-SCID chimeras.
(0.75 MB PDF)

Figure S5 Frequency of Vα24^+^Vβ11^+^ NKT cells. The frequency of immature and mature Vα24^+^Vβ11^+^ NKT cells in human fetal thymic cells as assessed by flow cytometry (**A**) and the ratio of rearranged Vα24-Jα18 and Cα DNAs in fetal thymocytes by Q-PCR (**B**) were examined before and after the positive depletion procedure [58], [59]. In **A**, thymic cells were stained with Vα24 and Vβ11 mAbs (left panels) or CD1d tetramer and TCRβ (right panels), respectively. Data were representative of three experiments or mean ± s.d. *, *p*<0.001.
(0.15 MB PDF)

Figure S6 The staining control data. For accurate quantitation of NKT cells, cells were stained with fluorochrome conjugated empty CD1d tetramers (eCD1d tetramer) and αβTCR isotype mAb (αβTCRIso) to establish the gate for negative controls. Cells were from the thymus and liver of EBV-exposed (**A**) or HTLV-1-exposed (**B**) hu-thy/liv-SCID chimeras at week 4 post-challenge as representatives for *in vivo* hu-thy/liv-SCID mouse experimental models. pt, post-transplantation. Other cells were from EBV-exposed RTOC (**C**) and FTOC (**D**) as representatives for *in vitro* experimental models.
(0.30 MB PDF)

Table S1 Clinical information of normal control and latent EBV-infected individuals, and patients with IM or HL.
(0.13 MB PDF)

Table S2 The absolute numbers of NKT cells and αβT cells (thymocytes) in different organs in various hu-thy/liv-SCID chimers.
(0.13 MB PDF)

Table S3 The sequences of primers and probes for mRNA and DNA detection in Q-PCR and Southern blot assays.
(0.11 MB PDF)
